RETRACTED

# Analysis of Interventional Application Effect of Ultrasound-Guided QLB and TAPB in the Treatment and Analgesia of Patients Undergoing Laparoscopic Colorectal Surgery

**DOI:** 10.1155/2022/4199868

**Published:** 2022-07-14

**Authors:** Zhengwei Chen, Yao Wang

**Affiliations:** ^1^Department of Gastrointestinal Surgery, Lishui City People's Hospital, Lishui 323000, China; ^2^Ultrasound Imaging Department of Lishui City People's Hospital, Lishui 323000, China

## Abstract

Colorectal cancer is a common malignant tumor of the digestive system. In order to study the clinical efficacy of ultrasound-guided QLB and TAPB in the treatment and postoperative analgesia of patients undergoing laparoscopic colorectal surgery. A total of 96 patients undergoing laparoscopic colorectal surgery from January 2021 to January 2022 are selected as the study subjects. The results show that ultrasound-guided QLB and TAPB therapy have good analgesic effects in patients undergoing laparoscopic colorectal surgery, and QLB treatment and postoperative analgesic effect are better than TAPB.

## 1. Introduction

Colorectal cancer is a common malignant tumor of the digestive system, and the incidence of cancer diseases is on the rise. With the continuous improvement of people's living standards, the incidence of this disease is also gradually increasing [1]. At the present stage, the clinical treatment of colorectal cancer is mainly through laparoscopic microincision, which has become a widely used surgical method in clinical practice due to its advantages of small wound, less intraoperative blood loss, and fast recovery [2, 3]. And intraoperative anesthesia is to ensure that the procedure would be able to give patients the basic conditions in order to alleviate patients' postoperative pain and intraoperative pain with strong stress response, to make patients achieve ideal anesthesia in the operation, and effective anesthesia can help patients with postoperative recovery and reduce the postoperative complications of [4, 5]. As one of the effective analgesic methods of anesthesia combined with multimode analgesia technology, TAPB block has achieved good analgesic effect in minimally invasive laparoscopic surgery, which can effectively relieve patients' body pain, but its deficiency is that it cannot be used as visceral analgesia [6, 7]. As one of the effective methods of postoperative multimode analgesia technology, ultrasound guided QLB block can improve the deficiency of TAPB and effectively relieve patients' visceral pain, which is widely used in gastrointestinal surgery, gynecological surgery, and other surgeries [8]. In order to study the treatment and analgesic effects of different blocking methods in laparoscopic colorectal surgery, this study analyzed and discussed the treatment and analgesic effects of patients undergoing laparoscopic colorectal surgery based on the ultrasound-guided QLB and TAPB blocking methods, in order to improve the reference for clinical treatment.

RETRACTED

The rest of this paper is organized as follows: Section 2 discusses relevant literature and comparative analysis, followed by the clinical treatment methods and evaluation indicators in Section 3. The comparative analysis and data statistics in Section 4.  Section 5 concludes the paper with a summary and future research directions.

## 2. Related Works

The disease of colorectal cancer develops rapidly and is induced by many reasons, such as: unhealthy eating habits, insufficient nutritional intake, and a low level of cellulose in the body. Surgical treatment is mainly used in clinic at the present stage [9, 10]. In order to relieve the pain of patients during and after surgery, general anesthesia combined with QLB block or TAPB block is performed during and after surgery, which has a significant effect on relieving the pain of patients [11, 12]. The mechanism of TAPB is to inject local anesthetic into the nerve fascia layer between the internal oblique muscle and transverse abdominis muscle to block relevant nerve sensory conduction so as to weaken the pain sensation in the skin, muscle, and parietal peritoneum of the anterior abdomen and achieve good abdominal analgesia [13, 14]. QLB can alleviate visceral pain and analgesia to a certain extent by blocking the somatic and sympathetic nerves in the thoracic paraspinal region. QLB can diffuse local anesthesia drugs from the psoas major and quadratus lumborum to the paraspinal, and the analgesic mechanism works faster. Meanwhile, it can inhibit abdominal visceral pain, which is beneficial to relieving stress response and stabilize intraoperative blood pressure and heart rate. TAPB anesthesia guided by ultrasound can improve the stress response and immune function of patients undergoing laparoscopic colon cancer surgery [15, 16]. The results of this study are basically consistent with the conclusion.

In addition, the results of this study show that after 10 minutes of skin cutting, HR of both groups increased, but the increase trend of the QLB group was lower than the TAPB group, and the change of blood pressure was relatively stable, so the QLB method could effectively stabilize the changes in HR and blood pressure of patients. COR and NK levels are compared between the two groups after surgery. The COR level in the QLB group is lower than that in the TAPB group, while the NK level in the QLB group is higher than that in the TAPB group. The stress response in both groups is effectively improved. However, the stress level in the QLB group is significantly reduced and the pain is effectively alleviated due to the TAPB group. Experimental results of relevant scholars show that the use of QLB in laparoscopic colorectal surgery can reduce intraoperative and postoperative drug consumption [17, 18]. The same conclusion is also reached in this study; the drug consumption of remifentanil and propofol in the two groups is lower in the QLB group than in the TAPB group. These results indicate that QLB has a better pain relief effect than the TAPB group in laparoscopic colorectal surgery. In addition, the results of this study also found that the estuation time of the QLB group is shorter than that of the TAPB group, and the first pressing time of the analgesia pump in the QLB group is longer than that of the TAPB group. The number of compressions of the analgesia pump in the QLB group was significantly less than that in the TAPB group, which also indicated that QLB had a better analgesic effect and had a longer block period than the TAPB group.

RETRACTED

In addition, the pain degree of the patients is also observed and recorded in this study. The results showed that the postoperative VAS scores of both groups are decreased, but the scores of the QLB group are significantly lower than that of the TAPB group, indicating that both the two block methods had good postoperative analgesia effect and could greatly reduce the pain symptoms of the patients. However, QLB block is more effective for postoperative analgesia. Other studies by relevant scholars show that QLB can effectively reduce the dosage during laparoscopic colorectal surgery, and the incidence of adverse reactions such as secondary nausea and vomiting and respiratory depression has also been significantly reduced [8, 19]. Using QLB block methods can provide more reliability than TAPB analgesia effect, also can reduce the incidence of complications. The conclusion of this study is consistent with that of scholars. In contrast, the study found that the dose, number of cases, incidence of nausea and vomiting, and remedial analgesia in QLB group and TAPB group were lower than those in TAPB group. These results proved that QLB block can provide a better block than TAPB and can also effectively reduce the incidence of nausea and vomiting and other adverse reactions [20]. In order to get the results and shortcomings of this study, only our hospital accepts cases as the research object, and the sample size selection range is small. As the research time is limited, selection of indicators is not comprehensive. For QLB block way to reduce the incidence of adverse reactions to the imperfection of the research, in the following study, each scholar can enlarge the sample size. Various indicators are selected to ensure that the research results are more comprehensive.

RETRACTED

## 3. Clinical Treatment Methods and Evaluation Indicators

### 3.1. Patients Information

A total of 96 patients undergoing laparoscopic colorectal surgery from January 2021 to January 2022 were selected as the study subjects. According to the random number table method, 96 patients were divided into two groups. In the QLB group (48 patients); there were 31 males and 17 females, with an average age of (41.42 ± 6.76) years. BMI ranged from 19 to 26 kg/m^2^, with an average of (23.4 ± 1.85) kg/m^2^. The other group was the TAPB group (48 persons). There were 27 males and 21 females, with an average age of (45.27 ± 5.16) years. The BMI ranged from 19 to 27 kg/m^2^, with an average of (24.4 ± 1.35) kg/m^2^. There are no significant differences in the two groups (*P* > 0.05), indicating comparability.

The inclusion criteria include the following aspects: (1) patient age >18 years old; (2) complete clinical data; (3) long-term analgesic drug users; (4) good understanding and communication skills; and (5) no history of mental illness.

The exclusion criteria include the following aspects: (1) local anesthetic allergy; (2) patients with serious heart disease; (3) abnormal liver and kidney function; (4) patients with coagulation dysfunction; and (5) infection in the puncture area.

All patients enrolled in the study signed informed consent, and the examination method and surgical method adopted in this study are clinically applied and safe methods. If they have any discomfort during treatment, they can inform their competent doctor in time to decide the next treatment plan. During the treatment, they are not allowed to use any other drugs or other disease treatment methods. If they use them, they must inform the doctor. In the process of this study, the original data (including test tables) belong to the research group. Patients have the right to privacy and their names will not appear in public publications. If relevant departments need it, they have the right to use these data. Patient participation is entirely voluntary. They have the right to choose not to participate in the study or withdraw from the study at any time. This does not affect the normal treatment of their disease, but they hope to complete this study without any special reasons.

### 3.2. Treatment Methods

The anesthesia methods include the following aspects: the same anesthesiologist performed anesthesia for patients in both groups. After entering the operating room, patients' vital signs such as heart rate, blood pressure, and oxygen saturation were monitored. Intravenous access is established after local anesthesia, and anesthesia is induced by anterior nerve block. Transverse abdominis block is performed in the TAPB group and quadratus lumborum block is performed in the QLB group. The blocking effect is measured by acupuncture 20 min later, and anesthesia is induced after satisfactory. Propofol 2.5 mg/kg, sufentanil 0.3 *μ*g/kg, and rocuronium 0.8 mg/kg are injected intravenously. After anesthesia induction, endotracheal intubation is performed, and anesthesia is maintained by intravenous anesthesia: remifentanil 0.3 *μ*g/(kg·min), propofol 6 mg/(kg·h), and cineatracurium 0.13 mg/(kg·h). Adjust anesthetic dosage according to HR, MAP, and BIS.

RETRACTED

The TAPB group includes the following aspects: a high-frequency ultrasound probe (6∼12 Hz, GE Healthcare Venue 50) is placed between the costal margin and the iliac crest, near the axillary front or midaxillary line, and three layers of abdominal external oblique muscle, internal oblique muscle, and transverse abdominis muscle are identified. The 22 G nerve block needle is placed in the transverse abdominal fascia from the outside to the inside of the plane, and then 2 mL of sterile normal saline is injected. After confirming the correct position of the needle tip, 20 mL of 0.37% is injected into the nerve fascia layer between the internal oblique muscle and the transverse abdominal muscle.

The QLB group includes the following aspects: the same ultrasonic instrument as the TAPB group is used, the probe frequency is adjusted to 3–5 MHz, and the probe is placed under the left costal margin and between the iliac crest. Transverse scanning is performed to reveal the vertebral bodies of L3 or L4, quadratus lumborum, psoas major, and erector spine muscles. The needle is inserted vertically at 3 cm beside the spinous process of L3 or L4. After the needle is inserted into the fascia space between the psoas major and quadratus lumborum, 1 mL 0.9% sodium chloride solution is injected for the water separation test. After the position of the tip is determined, another 25 ml 0.33% ropivacaine is injected according to the muscle stratification. Analgesic methods: After surgery, patients in both groups are given intravenous controlled analgesia (PCIA): sentinel is diluted to 100 mL with 100 *μ*g, the controlled analgesia is 0.5 ml, and the locking time is 15 min.

### 3.3. Observation Indicators and Evaluation Criteria

The observation indicators and evaluation criteria include the following aspects: (1) HR and blood pressure of the two groups are observed before and 10 minutes after skin excision; (2) postoperative stress response (COR and NK) is compared; (3) the dosage (remifentanil and propofol) of patients is compared; (4) time of postoperative estuation, time of first pressing analgesic pump, and time of pressing analgesic pump are compared; (5) visual analogue scale (VAS score) of pain in the two groups 1, 3, and 6 hours after surgery is compared. VAS score: 0 is no pain, 1–5 is mild pain, 5–9 is moderate pain, and more than 10 is severe pain. (6) Incidence of remedial analgesia, nausea and vomiting and confusion of consciousness.

RETRACTED

### 3.4. Statistical Processing

SPSS 25.0 statistical software is used for data analysis. Normality test is performed on the data first. Measurement data are expressed as (*x*‾±*s*). Paired sample *t* is used for test within the group, variance comparison is used between groups, and F test is performed for comparison between multiple groups. Repeated measurement is used between multiple groups to conduct spherical test. The count data include the following aspects: descriptive statistical analysis is conducted by percentage and *x*^2^ test is performed. *P* < 0.05 indicates significant difference.

## 4. Comparative Analysis and Data Statistics

### 4.1. Heart Rate and Blood Pressure are Observed

The heart rate of patients in both groups increased with skin excision, and the heart rate of patients in the QLB group is significantly lower than that of the TAPB group (*P* < 0.05), as shown in Table 1.

Blood pressure in both groups increased with the operation, and the QLB group was significantly lower than the TAPB group (*P* < 0.05), as shown in Table 2. In Table 2, “^*∗*^” indicates that compared with before sectioning.  Figure 1 is the comparison and analysis of hearth rate and blood pressure.

### 4.2. Comparison of Stress Response after Surgery

Compared with the TAPB group, COR level in the QLB group is significantly lower and NK expression is significantly higher (*P* < 0.05), as shown in Table 3.

### 4.3. Comparison of the Drug Dosage

The dosage of remifentanil and propofol in the QLB group is lower than that in the TAPB group (*P* < 0.05), as shown in Table 4.

### 4.4. Comparison of VAS Scores 1, 3, and 6 h after Surgery

The pain degree in both groups decreased over time, but the pain degree in QLB patients is significantly lower than that in patients of the TAPB group (*P* < 0.05), as shown in Table 5. In Table 5, “#” indicates compared with the later 1 h (# *P* < 0.05); “&” indicates compared with 3 h after surgery (& *P* < 0.05).

After surgery, VAS scores 1, 3, and 6 h are compared in Figure 2. In Figure 2, the “#” indicates significant difference in pain degree between the two groups in the same time period; “*a*, *b*, *c*, *d*” indicates that there is no difference if the letters are shared.

RETRACTED

### 4.5. Comparison of the Incidence of Adverse Reactions

The incidence of remedial analgesia and nausea and vomiting in the QLB group is lower than that in the TAPB group (*P* < 0.05), but there is no significant difference in the incidence of confusion, as shown in Table 6.

Figure 3 is the comparison of the incidence of adverse reactions.

## 5. Conclusion

In conclusion, ultrasound-guided application of QLB and TAPB blocks can alleviate the pain during the treatment and analgesia of patients undergoing laparoscopic colorectal surgery, and QLB is a new trunk nerve block method. Compared with TAPB block, QLB block can effectively reduce the number of anesthetics used during surgery. Moreover, the postoperative analgesia effect is superior to TAPB block, and the duration of action is longer than TAPB block, which can relieve postoperative stress reactions and reduce the occurrence of postoperative nausea and vomiting and other adverse reactions. It has good clinical effect in the treatment and analgesia of colorectal surgery patients and has clinical application value.

## Figures and Tables

**Figure 1:** Heart rate and blood pressure.

**Figure 2:** Comparison of VAS scores 1, 3, and 6h after surgery.

**Figure 3:** Comparison of the incidence of adverse reactions.

**Table 1:** Heart rate comparison.

Group	Number	Preoperative (times/min)	Peel for 10 minutes (times/min)	*t*	*P*
QLB group	48	64.13 ± 7.45	73.10 ± 7.11	1.418	0.002
TAPB group	48	65.36 ± 8.61	78.88 ± 8.75	2.145	0.011
*t*		2.474	3.014		
*P*		0.659	0.032		

**Table 2:** Blood pressure contrast.

	Group	SBP (mmHG)	DBP (mmHG)
Preoperative	QLB (*n* = 48)	90.08 ± 3.26	68.51 ± 4.25
	TAPB (*n* = 48)	89.36 ± 3.36	68.32 ± 4.56

	*t*	2.412	1.471
	*P*	0.061	0.464
Peel for 10 minutes	QLB (*n* = 48)	102.03 ± 4.56^*∗*^	75.06 ± 4.02^*∗*^
	TAPB (*n* = 48)	109.06 ± 4.32^*∗*^	79.15 ± 3.59^*∗*^

	*t*	2.964	2.454
	*P*	0.041	0.012

**Table 3:** Stress response after surgery.

Group	Number	COR (nmol/L)	NK (%)
QLB group	48	451.85 ± 90.03	22.43 ± 3.04
TAPB group	48	510.14 ± 88.62	17.17 ± 2.59
*t*		2.657	3.321
*P*		0.016	0.022

**Table 4:** The drug dosage.

Group	Number	Remifentanil [*μ*g/(kg·min)]	Propofol [mg/(kg·h)]
QLB group	48	0.15 ± 0.02	5.42 ± 1.01
TAPB group	48	0.19 ± 0.03	5.71 ± 1.04
*t*		0.541	0.965
*P*		0.036	0.024

**Table 5:** Comparison of VAS scores 1, 3, and 6 h after surgery.

Group	Number	Before the surgery	1 h after the surgery	3 h after the surgery	6 h after the surgery	*F*	*P*
QLB group	48	6.27 ± 1.29	3.35 ± 0.12^*∗*^	2.21 ± 0.24^*∗*^^#^	1.32 ± 0.04^*∗*^^#&^	0.747	0.015
TAPB group	48	6.21 ± 1.27	4.57 ± 0.24^*∗*^	3.13 ± 0.27^*∗*^^#^	2.03 ± 0.17^*∗*^^#&^	1.447	0.022
*t*		0.321	0.476	0.853	0.412		
*P*		0.617	0.043	0.026	0.003		

RETRACTED

**Table 6:** Comparison of the incidence of adverse reactions.

Group	Number	Remedial analgesia (%)	Nausea and vomiting (%)	Blurred consciousness (%)
QLB group	48	3 (6.25)	5 (10.42)	1 (2.08)
TAPB group	48	8 (16.67)	11 (22.92)	2 (4.17)
*x* ^2^		2.668	2.774	1.363
*P*		0.004	0.001	0.052

## Data Availability

The simulation experiment data used to support the findings of this study are available from the corresponding author upon request.
